# Identification of immune-related lncRNAs to improve the prognosis prediction for patients with papillary thyroid cancer

**DOI:** 10.1042/BSR20204086

**Published:** 2021-02-23

**Authors:** Zhiyang Li, Weixun Lin, Jiehua Zheng, Weida Hong, Juan Zou, Taofeng Zhang, Yexi Chen, Hai Lu

**Affiliations:** 1 The Second Affiliated Hospital of GuangZhou University of Chinese Medicine, Guangzhou, Guangdong Province 510282, P.R. China; 2 The Second Clinical College of Guangzhou University of Chinese Medicine, Guangzhou, Guangdong Province 510282, P.R. China; 3 Department of Thyroid, Breast and Hernia Surgery, The Second Affiliated Hospital of Shantou University Medical College, Shantou, Guangdong 515041, P.R. China

**Keywords:** ceRNA network, immune-related lncRNA, papillary thyroid cancer, PD1

## Abstract

Objective: To identify immune-related long non-coding RNAs (lncRNAs) in papillary thyroid cancer (PTC).

Methods: The Gene Expression Omnibus (GEO) and The Cancer Genome Atlas (TCGA) databases were used to obtain the gene expression profile. Immune-related lncRNAs were screened from the Molecular Signatures Database v4.0 (MsigDB). We performed a survival analysis of critical lncRNAs. Further, the function of prognostic lncRNAs was inferred using the Gene Ontology (GO) enrichment analysis and Kyoto Encyclopedia of Genes and Genomes (KEGG) to clarify the possible mechanisms underlying their predictive ability. The assessment was performed in clinical samples and PTC cells.

Results: We obtained 4 immune-related lncRNAs, 15 microRNAs (miRNAs), and 375 mRNAs as the key mediators in the pathophysiological processes of PTC from the GEO database. Further, Lasso regression analysis identified seven prognostic markers (LINC02550, SLC26A4-AS1, ACVR2B-AS1, AC005479.2, LINC02454, and AL136366.1), most of which were related to tumor development. The KEGG pathway enrichment analysis showed different, changed genes mainly enriched in the cancer-related pathways, PI3K-Akt signaling pathway, and focal adhesion. Only SLC26A4-AS1 had an intersection in the results of the two databases.

Conclusion: LncRNA SLC26A4-AS1, which is the most associated with prognosis, may play an oncogenic role in the development of PTC.

## Introduction

Papillary thyroid cancer (PTC) is the most common type of thyroid cancer. PTC accounts for approximately 80% of all thyroid cancers [1]. Although PTC generally has a good prognosis, tumor recurrence and metastasis impede clinical management and individual patient survival [2]. Therefore, further understanding of the molecular mechanism of PTC to develop effective methods for early screening and diagnosis is critical for reducing the number of PTC patients who are not diagnosed before the onset of aggressive disease.

Long non-coding RNAs (lncRNAs), which do not have protein-coding functions, have recently attracted increasing research attention [3]. These RNAs play a significant role in different cellular processes, particularly in numerous tumors [4]. MicroRNAs (miRNAs) are small, endogenous, non-coding RNAs composed of 19–25 nucleotides. They exert the critical function of regulating gene expression, and their regulatory networks are involved in many biological processes [5]. Previous studies on the competing endogenous RNA (ceRNA) have focused on the mechanism hypothesis, presented by Salmena et al., which has been described as the ‘Rosetta Stone’ for decoding the RNA language used in regulating RNA cross-talk and modulating biological functions [6]. The core concept is that ceRNAs interact with target miRNAs through miRNA response elements to control the transcriptome on a large scale. Recently, an increasing number of lncRNAs have been discovered in the tumorigenesis of PTC. For example, Feng et al. found that lncRNA n384546 promotes PTC progression and metastasis [7]. However, previous studies have focused on the mechanism of a single lncRNA–miRNA–mRNA axis, and there is currently no reported ceRNA network in PTC. Consequently, it is imperative to investigate the role of ceRNA networks in the poor prognosis of PTC. By further learning how lncRNAs function in the pathogenesis of PTC, we may find solutions to the most pressing challenges faced while treating this disease.

Immunotherapy is another promising approach for overcoming the poor prognosis of PTC patients after standard therapy and restricted applicability of targeted therapies. Currently, several immune-related parameters, mainly tumor-infiltrating lymphocytes, have been reported to predict the prognosis of cancer patients, suggesting that immune states have a significant impact on the prognosis of patients [8]. Therefore, it is necessary to systematically study immune-related lncRNAs in the PTC microenvironment to understand the complex anti-tumor response better and determine effective immunotherapy for PTC.

In the present study, we constructed a ceRNA regulatory network to determine how immune-related lncRNAs act as a sponge for miRNA to regulate PTC gene expression. We found that immune-related lncRNA SLC26A4-AS1, which is the most associated with disease-free survival, may play an oncogenic role in the development of PTC. The present study might provide an insight into the molecular mechanisms that participate in progression and tumorigenesis of PTC.

## Materials and methods

### Data collection and processing

We searched the Gene Expression Omnibus (GEO) database (www.ncbi.nlm.nih.gov/geo/) and The Cancer Genome Atlas (TCGA) data portal (https://cancergenome.nih.gov/). We used the following search terms: papillary thyroid carcinoma and PTC. We obtained data from GEO for 64 PTC samples and 61 normal thyroid tissue samples (GSE33630, GSE3467, and GSE3678) and TCGA, which contained data from 493 primary PTC samples and 58 non-tumor tissues. Furthermore, we downloaded 319 lncRNAs related to the immune system process M13664, immune response M19817, immune effector process M14818, immune system development, and the M3457 pathway from the Molecular Signatures Database (MSigDB;https://www.gsea-msigdb.org/gsea/msigdb).

### Construction of the lncRNA–miRNA–mRNA network of PTC

We analyzed the gene expression data using the DESeq2 package and ggplot2 package of R software for each group and sample. Reverse-transcription quantitative PCR was used to identify common differentially expressed genes (DEGs) from the datasets, and they were integrated using Venn analysis. We obtained the miRNA sequences from the StarBase database (http://starbase.sysu.edu.cn/). MiRcode (http://www.mircode.org/) [9] is an effective online software that provides the interactions between lncRNAs and miRNAs. MiRTarBase (http://mirtarbase.mbc.nctu.edu.tw) [10], miRDB (http://www.mirdb.org/miRDB/) [11], and TargetScan (http://www.targetscan.org/) [12] are online tools that were used to retrieve and predict target mRNAs of the miRNAs. A Venn diagram was constructed to obtain the overlapping portion of target miRNAs and mRNAs.

### Analysis of immune characteristics between the high- and low-risk groups

We used a multivariate Cox regression model to screen immune-related lncRNAs. After incorporating the expression levels of specific genes, each patient’s risk score formula was constructed and weighted by its estimated regression coefficient. According to the risk score formula, patients were divided into the low- and high-risk groups with the median risk score as the cut-off point.

### Functional and survival analysis

We used the clusterprofiler package of R software to perform Gene Ontology (GO) function analysis and Kyoto Encyclopedia of Genes and Genomes (KEGG) pathway analysis of the above common DEGs. *P*<0.05 was used as a threshold to screen significant enrichment functions and pathways. The lncRNAs in the PTC lncRNA–miRNA–mRNA network were identified as crucial lncRNAs. LncRNA correlations with patient survival were featured in GEPIA for Kaplan–Meier survival analysis.

### Tissues sample collection and total RNA extraction

We collected a total of 10 PTC tissue samples and 20 normal tissue samples from patients who underwent surgery between 2018 and 2019 at the Second Affiliated Hospital of Shantou University (Guangdong, China). The Ethics Committee approved the present study at the Second Affiliated Hospital of Shantou University (Guangdong, China), and all patients provided written informed consent. Following resection, the tissues were immediately frozen at −80°C. TRIzol reagent (Invitrogen; Thermo Fisher Scientific, Inc.) was used to extract the total RNA from PTC cells and tissue samples.

### Reverse-transcription quantitative PCR

*In vitro*, we mixed the cultured cells and plasma with TRIzol reagent (Invitrogen, U.S.A.) to extract total RNA. Tumor tissues and adjacent healthy tissues were ground in liquid nitrogen before the addition of TRIzol reagent. Reverse transcription was performed using RNA samples as a template to synthesize cDNA. We used SYBR Green Real-Time PCR Master Mix (Thermo Fisher Scientific, U.S.A.) to prepare the PCR system.

### Cell culture and transfection

Human PTC cell lines IHH-4 and HTH83 were provided by the American Type Culture Collection (ATCC, U.S.A.). Cells were cultured in DMEM containing 10% FBS (Invitrogen, Carlsbad, CA, U.S.A.), 100 U/ml streptomycin (Invitrogen, Carlsbad, CA, U.S.A.), and 100 mg/ml penicillin G (Invitrogen, Carlsbad, CA, U.S.A.) in an incubator (37°C, 5% CO_2_). Cells were collected during the logarithmic growth phase for subsequent experiments. We transfected cells with 50 nM negative control (NC) or SLC26A4-AS1 small interfering (si) RNA using Lipofectamine RNAi MAX reagent (Thermo Fisher Scientific, Inc.). After 24 h of transfection, subsequent experiments were performed.

### Cell migration and proliferation assay

Following transfection, cells were resuspended in RPMI medium without FBS at a density of 2 × 10^4^ cells/well. We seeded a total of 100 μl resuspended cells into the upper chamber of a Transwell insert. RPMI medium supplemented with 10% FBS was added to the lower chamber. The cells were cultured at 37°C with 5% CO_2_ for 25 h. Migratory cells were fixed in 70% paraformaldehyde for 30 min and stained with 0.1% Crystal Violet for an additional 30 min at room temperature. After being washed with PBS, cells were directly observed using an inverted microscope and were counted in five randomly selected fields to obtain the average using ImageJ (version 1.48; National Institutes of Health). Following transfection, IHH-4 and HTH83 cells were seeded into 96-well plates at a density of 5 × 10^3^ cells/well. At the 24, 48, 72, and 96 h time points, 101 Cell Counting Kit-8 (CCK-8; Dojindo Molecular Technologies, Inc.) solution was added to each well, and the plates were incubated at 37°C for 1 h in the dark. Absorbance was measured at a wavelength of 450 nm using a microplate reader.

### Cells detected by flow cytometry

Cells were washed twice with cold PBS and binding buffer was added (100 µl). Cells were incubated with PE-Annexin V (5 µl) and 7AAD (5 µl) for 15 min in the dark at room temperature. Cells were washed with fresh binding buffer, then 400 µl of binding buffer were added to the cells, re-suspended and analyzed in an Agilent NovoCyte Quanteon flow cytometer (Agilent Technologies Co. Ltd, U.S.A.). The fluorescence was quantified by CSampler software (Becton, Dickinson and Company, Franklin Lakes, NJ, U.S.A.).

## Results

### Establish PTC’s lncRNA–miRNA–mRNA ceRNA network

The GSE3678, GSE3467, and GSE33630 databases had 64 PTC samples and 61 paired normal thyroid tissue samples. The TCGA database had 493 primary PTC samples and 58 non-tumor tissues. Following data processing using the LIMMA package, 1189, 1194, and 2226 DEGs were extracted from the expression profile datasets GSE3678, GSE3467, and GSE33630, respectively (Figure 1A–D). After screening out immune-related lncRNAs, we finally obtained four lncRNAs, which were identified by Venn analysis (Figure 1E). Hierarchical clustering of the identified DEGs is displayed as a heatmap in Figure 1F. We obtained 96 abnormally expressed miRNAs significantly relevant to PTC survival from OncomiR. Four PTC-specific lncRNAs putatively interacted with 15 PTC-specific miRNAs. Then, the relationships between cancer-specific miRNAs and cancer-specific mRNAs were evaluated. A total of 435 PTC-specific mRNAs targeted by 25 PTC-specific miRNAs were identified. Based on the above data, the lncRNA–miRNA–mRNA ceRNA network of PTC (Figure 2) was established and plotted using Cytoscape 3.7.0.

**Figure 1:** Gene expression of each dataset (**A–C**) A volcano graph displaying pairs of expressed genes. Red dots indicate significantly up-regulated DEGs, and blue dots indicate significantly down-regulated DEGs that passed the screening threshold. (**D**) DEG counts of each dataset. (**E**) Venn analysis among DEGs of three datasets. (**F**) Heatmap and hierarchical clustering of identified DEGs. Up- or down-regulated genes are colored in red or blue, respectively.

**Figure 2:** The immune-related lncRNA–miRNA–mRNA ceRNA network in PTC The hexagon represents cancer-specific lncRNA. The octagon represents cancer-specific miRNA. The ellipse represents cancer-specific mRNA.

### Immune-related lncRNA was significantly related to the prognosis of PTC

The PTC patients were divided into two groups based on the Lasso analysis. There were significant differences in clinical outcomes for overall survival (OS) between the two groups of patients. Figure 3 shows a heat map of the included immune-related lncRNA expression profile (Figure 3A) and K–M analysis of the significant difference in survival between the two groups (Figure 3B).

**Figure 3:** Immune-related lncRNAs in PTC from TCGA (**A**) Heat map of the expression profile of the included immune-related lncRNA. (**B**) Patients in the high-risk group have a shorter OS.

### The main pathways regulated by lncRNA

We analyzed lncRNA-regulated GO terms (Figure 4A–C). In the PTC lncRNA–miRNA–mRNA ceRNA network, the result showed that the mRNAs related to the biological process were most relevant to signal transduction. mRNAs related to the cellular component were most relevant to the integral component of the membrane, and molecular function was most relevant to calcium ion binding. We performed pathway enrichment analysis of the mRNAs of the lncRNA–miRNA–mRNA ceRNA network and identified the lncRNA regulated pathway (Figure 4D). Functional analysis showed the top three lncRNA regulated pathways were pathways in cancer, the PI3K-Akt signaling pathway, and focal adhesion. We used GEPIA to perform survival analysis of prognosis-related lncRNAs (Figure 5). Only SLC26A4-AS1 had an intersection in the results of the two databases. Similarly, only SLC26A4-AS1 was significantly associated with disease-free survival in GEPIA.

**Figure 4:** GO analysis and KEGG analysis in the ceRNA network (**A–C**) GO analysis of mRNAs in the ceRNA network. x-axis reflects the gene count; y-axis reflects different GO terms. The column color reflects the *P*-value (−log10(*P*-value)): black represents the biggest value; blue represents the smallest value. (**D**) The node size reflects the gene count: the bigger the gene count, the bigger the node size. The node color reflects the *P*-value (−log10(*P*-value)): the bigger the −log10(*P*-value) value, the darker the node color.

**Figure 5:** Analyses of clinical prognosis of SLC26A4-AS1 (**A**) Analyses of SLC26A4-AS1 expression in tumor vs. normal tissues and different tumor stages. (**B**) Overall and disease-free survival analyses of SLC26A4-AS1. (A) Analyses of pivotal lncRNA expression in tumor vs. normal tissues and different tumor stages. The red box represents tumor tissue; the gray box represents normal tissue; dots represent each sample value. *P<0.05; other *P*-values are shown on the diagrams. (B) Overall and disease-free survival analyses of hub lncRNAs. *P*-values are shown in the diagrams.

### Silencing of SLC26A4-AS1 inhibited IHH-4 and HTH83 cells growth

SLC26A4-AS1 expression levels were detected in normal tissues (*n*=10) and PTC tissues (*n*=20). The results revealed that the expression levels of SLC26A4-AS1 were significantly increased in PTC tissues (*P*=0.0090; Figure 6A). To further investigate the functions of SLC26A4-AS1, siRNA targeting SLC26A4-AS1 was established and knockdown assays were subsequently performed *in vitro*. Transfection efficiency is illustrated in Figure 6B, and the SLC26A4-AS1 group exhibited significantly decreased levels of SLC26A4-AS1 compared with the control group in both the cell lines tested. The results of the CCK-8 assay revealed that cell proliferation was significantly inhibited following SLC26A4-AS1 knockdown (Figure 6C,D). In addition, results from Transwell assays showed that migration was significantly abrogated in IHH-4 and HTH83 cells following SLC26A4-AS1 knockdown (Figure 6E,F).

**Figure 6:** SLC26A4-AS1 promotes proliferation and migration in PTC cells *in vitro* (**A**) SLC26A4-AS1 levels were higher in PTC samples compared with normal tissues. (**B**) siRNA transfection efficiency. (**C**) Cell proliferation was measured using a CCK-8 assay in IHH-4 and (**D**) HTH83 cells following SLC26A4-AS1 silencing. (**E**) Cell migration was measured by Transwell assay in IHH-4 and (**F**) HTH83 cells following SLC26A4-AS1 silencing (magnification, ×200). **P<0.01.

### Overexpression of SLC26A4-AS1 inhibited the function of immune cells in PTC patients

As shown in Figure 7A, co-culture with IHH-4 cells, which were transfected with SLC26A4-AS1, resulted in reduction in proliferation of CD8^+^ T cells, but this phenomenon could be partly relieved by administration of the anti-PD-L1 antibody. NK cells normally do not express PD-1, but after culture in the IHH-4 derived condition medium+IL-15, PD-1 expression was noted on the surface of NK cells. These PD-1+NK cells were used in cytotoxicity assay. As shown in Figure 7B, IHH-4 cells were pre-stained with CFSE, and they served as the target cells for NK cells. The cytotoxicity of PD-1+NK cells was decreased after IHH-4 cells were transfected with SLC26A4-AS1, but this phenomenon could be partly relieved by administration of the anti-PD-L1 antibody. As shown in Figure 7C, after co-culture with IHH-4 cells, which were transfected with SLC26A4-AS1, the apoptosis rate of T cells was significantly enhanced compared with that in the control group, and this phenomenon could be partly relieved by administration of the anti-PD-L1 antibody. This result indicated that the immune-suppression function of SLC26A4-AS1 is dependent on PD-L1 expression. Taken together, our results indicated that SLC26A4-AS1 overexpression in PTC suppresses the immune cell function.

**Figure 7:** SLC26A4-AS1 overexpression in PTC suppresses the immune cell function (**A**) CFSE was used to evaluate the proliferation of T cells. T cells were cultured directly with IHH-4 cells transfected with SLC26A4-AS1 or not for 48 h, and the column shows the percentage of T cells. (**B**) NK cell cytotoxicity assay was performed, IHH-4-CFSE, which were transfected with SLC26A4-AS1 or not, were used as the target cells. (**C**) T cells were cultured directly with IHH-4 cells transfected with SLC26A4-AS1 or not for 48 h. The apoptosis rate was evaluated by Annexin V staining.

## Discussion

Over the last few years, the ceRNA hypothesis has been considered a novel layer of gene regulation. Our knowledge about the molecular mechanism of lncRNA in cancer is still limited. In the present study, we identified cancer-specific lncRNAs, miRNAs, and mRNAs in PTC. According to the bioinformatics differential analysis, we constructed a ceRNA network. We predicted functions of DEGs in PTC by the GO and pathway analyses. Of the genes involved in the ceRNA network, KEGG analysis showed that these genes were mainly enriched in two pathways related to cancer: pathways in cancer and the PI3K-Akt signaling pathway. There was evidence that the PI3K-Akt signaling pathway plays an essential role in PTC tumorigenesis. Hao et al.’s study showed that the PI3K-Akt signaling pathway activation was associated with PTC cell proliferation, migration, and invasion [13]. Zheng et al. found that TEKT4 promoted PTC cell metastasis through activating the PI3K/Akt pathway [14]. The regulation function of lncRNAs through the PI3K/Akt pathway in PTC is worthy of study. The ceRNA network identified in our analysis provided useful clues for further research.

Among the immune-related lncRNAs from the GEO database analysis, SLC26A4-AS1 is associated with PTC disease-free survival. LncRNA NR2F1-AS1 is broadly expressed in the brain [15], gall bladder [16], and other tissues. TNRC6C-AS1 is broadly expressed in lymph nodes [17], spleen [18], and other tissues. LOC646736 is restrictedly expressed in the thyroid [19]. Further molecular biological experiments are needed to confirm the function of the identified genes.

We found that only SLC26A4-AS1 had an intersection in the results of the two databases. Similarly, only SLC26A4-AS1 was significantly associated with disease-free survival in GEPIA. The expression levels of SLC26A4-AS1 were determined in PTC clinical samples using RT-qPCR. The results revealed that SLC26A4-AS1 was highly expressed in PTC tissues compared with normal tissue samples. Functional cell-based assays further confirmed that SLC26A4-AS1 played a role in the proliferation and migration of IHH-4 and HTH83 cells. The PD-L1 axis is a classical checkpoint that induces an immune-suppression effect in T cells. In the present study, we confirmed that SLC26A4-AS1 overexpression-induced up-regulation of PD-L1 could enhance T-cell apoptosis and restrict T-cell proliferation. Li et al. reported that PD-1 expression in NK cells was induced when incubated with tumor cells [20]. In this study, the cytotoxicity of PD-1+NK cells could be impaired by PD-L1 up-regulation induced by SLC26A4-AS1 overexpression in PTC cells. To further examine the mechanism of SLC26A4-AS1, RNA immunoprecipitation and chromatin immunoprecipitation assays will be performed in future studies.

In our study, we identified four immune-related lncRNAs from the GEO database and six immune-related lncRNAs from the TCGA database. Finally, we determined that SLC26A4-AS1 was the most prognostic immune-related lncRNA. It is meaningful to explore new biomarkers for diagnosis, prognostication, and PTC therapeutic targets to develop more effective surveillance and treatment programs. The present study provides the right direction for further research. Functional studies that can further delineate the biologic basis of PTC are needed.

## Conclusion

We constructed a PTC-specific ceRNA network and chose four hub lncRNAs for PTC by bioinformatics analysis. We described a method for identifying the potential lncRNA biomarkers. We found that SLC26A4-AS1, which is most associated with disease-free survival, may play an oncogenic role in the development of PTC. Furthermore, we found the ceRNA network in PTC, which should help to further our understanding of the mechanism underlying the pathogenesis of this disease.

## Data Availability

Data can be obtained from the corresponding author.

## Abbreviations

CCK-8: cell counting kit-8
ceRNA: competing endogenous RNA
DEG: differentially expressed gene
GEO: Gene Expression Omnibus
GO: Gene Ontology
KEGG: Kyoto Encyclopedia of Genes and Genomes
lncRNA: long non-coding RNA
miRNA: microRNA
MSigDB: Molecular Signatures Database
NK: natural killer
OS: overall survival
PD-1: programmed death receptor 1
PD-L: programmed cell death-ligand 1
PTC: papillary thyroid cancer
RT-qPCR: real time quantitative reverse transcription
TCGA: The Cancer Genome Atlas
